The article "Forecast of E-Commerce Transactions Trend Using Integration of Enhanced Whale Optimization Algorithm and Support Vector Machine" was published in 2021. Journal: Comput Intell Neurosci.

# Forecast of E-Commerce Transactions Trend Using Integration of Enhanced Whale Optimization Algorithm and Support Vector Machine

**DOI:** 10.1155/2021/9931521

**Published:** 2021-07-19

**Authors:** Suqi Zhang, Hsiung-Cheng Lin, Xinxin Wang

**Affiliations:** ^1^School of Information Engineering, Tianjin University of Commerce, Tianjin 300134, China; ^2^Department of Electronic Engineering, National Chin-yi University of Technology, Taichung 41170, Taiwan; ^3^School of Science, Tianjin University of Commerce, Tianjin 300134, China

## Abstract

E-commerce has become a crucial business model through the Internet around the world. Therefore, its transaction trend forecast can provide important information for the market planning and development in advance. For this purpose, the integrated model of enhanced whale optimization algorithm (EWOA) with support vector machine (SVM) is proposed for forecast of E-commerce transaction trend in this study. First, the global optimization ability of the whale optimization algorithm (WOA) is enhanced by the search updating strategy. Second, multiple factors that may affect the E-commerce transaction trend are analyzed and determined using the gray correlation mechanism. Third, the EWOA algorithm is employed to optimize the SVM random parameters. Finally, the EWOA-SVM model is established for forecasting E-commerce transaction trend. Two representative cases tests confirm that the EWOA-SVM model is superior to other existing methods in terms of fast convergence speed and high prediction accuracy.

## 1. Introduction

The current digital economy is moving forward much faster than before in recent years. Therefore, E-commerce transactions have become an important core of the digital economy in the global market [1, 2]. The rapid E-commerce development has resulted in certain changes in the logistics, manufacturing and traditional retail industries, etc. Transaction volume is usually regarded as a crucial indicator used for assessment of the E-commerce development level. As a result, E-commerce transactions trend forecast is indispensable to provide a quantitative basis for the long-term planning and strategy formulation for enterprises and governments [3, 4].

At present, the prediction methods applied for E-commerce transactions trend have been focused on machine learning models, regression models, and combination models [5, 6]. Machine learning models include neural network model, support vector machine (SVM), extreme learning machine (ELM), etc. [7]. They are somehow sensitive to parameters selection to predict the E-commerce transactions trend through the mapping relationship between influencing factors and transactions volume [8]. The regression models mainly refer to moving average model (MA), autoregressive model (AR), autoregressive moving average model (ARMA), and the nonlinear regression models. They may work well in analyzing the stationary series, but they are not suitable for the nonstationary time series analysis. On the other hand, the combination models can provide competitive results and outperform the single model, but their computational cost is relatively higher than that of the single model [9, 10].

Zhang et al. [11] applied the ELM model for forecasting E-commerce transactions and proposed an improved optimization algorithm to optimize the random model parameters. However, only few basic influencing factors were considered so that it may be not applicable in real circumstances. Ji et al. [12] combined XGBoost and ARIMA models to predict the size of E-commerce transactions, presenting better results than individual XGBoost and ARIMA models, but the complexity and computational cost may post a difficulty for further applications. Alternatively, Chen et al. [13] combined clustering technology and machine learning model to forecast the transaction size. Clustering technology is used to divide the training samples, and then the machine learning model was applied to train groups. The random parameters that may influence machine learning performance were not well considered, resulting in the instability of prediction results. Di Pillo et al. [14] employed SVM to predict the sales scale. Compared with linear regression models, the SVM model has a stronger nonlinear mapping ability. However, it is sensitive to random model parameters. Mao et al. [15] predicted China's E-commerce online transaction volume based on the combination of ARMA model and gray model, and the forecasting result was satisfactory.

SVM model is suitable for small sample prediction, and it has strong generalization ability and less random parameters. Li et al. [16] proposed an improved dragonfly algorithm to optimize SVM's random parameters in short-term wind power prediction. Liu et al. [17] applied SVM to forecast the remaining life of lithium-ion batteries and used chicken swarm optimization algorithm to solve random parameters. Pham et al. [18] employed the SVM model for rainfall prediction and achieved high prediction accuracy. Additionally, Hossain and Muhammad [19] applied SVM in emotion recognition system for emotion classification. Huang and Wang [20] used SVM model for pattern classification, where the genetic algorithm was applied to optimize model's random parameters to improve classification accuracy.

For SVM to be used for forecasting the E-commerce transaction trend, two main problems need to be resolved. The first task is to reduce the influence of random parameters of SVM model, which is an optimization point. The other is to choose crucial factors on E-commerce transaction trend. Consequently, this study proposes an integrated model using enhanced Whale Optimization Algorithm (EWOA) with SVM model on the basis of multiple factors analysis and machine learning. In this approach, EWOA algorithm was used to optimize the random parameters of SVM model. The modeling process is introduced in Section 2.  Section 3 analyzes multiple influencing factors and determines critical points on E-commerce transactions.  Section 4 validates the proposed model through two cases. The conclusions with future work are presented in Section 5.

## 2. Models of E-Commerce Transaction Trend Forecast

### 2.1. SVM Model

SVM, which is a hot spot model in machine learning models, has the characteristics of simple structure, few adjustable parameters, and strong generalization ability. It is often used in pattern recognition, disease diagnosis, regression prediction, and other fields [21]. The samples are mapped to the high-dimensional space *R*^*N*^ through a mapping function *φ*(*x*). Given a sample set {(*x*_*i*_, *y*_*i*_)*|x*_*i*_ ∈ *R*^*N*^, *y*_*i*_ ∈ *R*,  *j*=1,2,…, *n*}, the hyperplane *g* between input *x* and output *y* is established in a high-dimensional space as follows [22]:

(1) $$\begin{array}{c} g\left(x\right)=w\cdot \varphi \left(x\right)+l,\;\left(w\in R^{N},l\in R\right), \end{array}$$

where *g*(*x*) represents the output function, *w* is the weight, and *l* indicates the offset.

*g*(*x*) is transformed into a constrained optimization problem through the principle of structural risk minimization. Taking into account the errors, the slack variable is introduced into the objective function. The constraints minimization is expressed as follows [23]:

(2) $$\begin{array}{c} \min\frac{1}{2}{\left\|w\right\|}^{2}+\rho \sum_{i=1}^{n}\left(\zeta_{i}+\zeta_{i}^{*}\right),\\ \left\{\begin{array}{c} y_{i}-l-w\cdot x_{i}\leq \tau +\zeta_{i},\\ l+w\cdot x_{i}-y_{i}\leq \tau +\zeta_{i}^{*},\\ \zeta_{i}^{*}\geq 0,\\ \zeta_{i}\geq 0, \end{array}\right. \end{array}$$

where *ζ*_*i*_ and *ζ*_*i*_^*∗*^ are slack variables, *ρ* is a penalty coefficient, and *τ* is the error.

The optimization problem is transformed into solving the equation by Lagrange multiplier, then the derivation of each variable is performed, and finally the dual form of the optimal problem is obtained [24, 25].

(3) $$\begin{array}{c} \left\{\begin{array}{c} \min\frac{1}{2}\sum_{i,j=1}^{n}\left(\alpha_{i}^{\wedge }-\alpha_{i}\right)\left(\alpha_{j}^{\wedge }-\alpha_{j}\right)\kappa \left(x_{i}\cdot x_{j}\right)+\tau \sum_{i=1}^{n}\left(\alpha_{i}^{\wedge }-\alpha_{i}\right)-\sum_{i=1}^{n}y_{i}\left(\alpha_{i}^{\wedge }-\alpha_{i}\right)\\ \sum_{i=1}^{n}\left(\alpha_{i}^{\wedge }-\alpha_{i}\right)=0\\ \alpha_{i}^{\wedge },\alpha_{i}\geq 0,\;\;i=1,2,3,\ldots ,n, \end{array}\right. \end{array}$$

where *α*_*i*_^∧^ and _*α*_^*i*^ are Lagrange multipliers, *κ*(*x*_*i*_ · *x*_*j*_) is kernel functions, and the radial basis function (RBF) kernel is used in this study.

(4) $$\begin{array}{c} \kappa \left(x_{i},x_{j}\right)=e^{-\left({\left\|x_{i}-x_{j}\right\|}^{2}/2\delta^{2}\right)}, \end{array}$$

where *δ* (*δ* > 0) is the size of the kernel parameter.

Finally, the SVM regression function is defined as follows:

(5) $$\begin{array}{c} g\left(x\right)=\sum_{i=1}^{n}\left(\alpha_{i}-\alpha_{i}{}^{⌃}\right)\kappa \left(x_{i},x_{j}\right)+l. \end{array}$$

Generally, in SVM model, the penalty coefficient *ρ* and kernel coefficient *δ* are random parameters, which bring uncertainty to the prediction results under the complexity of the data. To solve this problem, these random parameters need to be optimized. For this reason, a whale optimization algorithm based on search updating strategy is proposed to optimize SVM parameters and achieve the prediction accuracy for E-commerce transaction trend.

### 2.2. WOA Algorithm

To date, a variety of intelligent algorithms have been developed and applied, such as PSO algorithm [26], crow search algorithm (CSA) [27], and a series of hybrid swarm algorithms [28–33]. Each algorithm uses a different method or strategy to fit some specific purposes or applications. For example, Zapata et al. [34] developed a hybrid swarm algorithm for collective construction of 3D structures, and Precup [35] proposed slime mould algorithm-based tuning of cost-effective fuzzy controllers for servo systems. Alternatively, WOA, which has a strong optimization ability, is a new swarm intelligence optimization algorithm [36]. It can simulate the predatory behavior of whales in nature, including foraging, encircling, bubble hunting, and food searching [37]. During the foraging phase, the information is exchanged between individuals in the whale group, and the food location is determined through the information communication. Usually, the initial optimal target position is used as the food position, and the whale can approach the food by updating its position. The whale location update strategy is described as follows [38, 39]:

(6) $$\begin{array}{c} x\left(m+1\right)=x\wedge \left(m\right)-A•B, \end{array}$$

(7) $$\begin{array}{c} B=\left|C•x\wedge \left(m\right)-x\left(m\right)\right|, \end{array}$$

where *m* is the current iteration number; **A** and **C** are coefficient matrices; **B** represents the distance between the whale and the food; **x** is the whale position, and **x**∧ represents the optimal position in the whale group.

The coefficient matrices **A** and **C** in equations (6) and (7) are calculated as follows:

(8) $$\begin{array}{c} A=2a•u-a,\\ C=2u, \end{array}$$

where **u** is a random number between 0 and 1; **a** decreases linearly from 2 to 0 in the iterative process.

The whales adopt enveloping and spiraling behaviors in the predation stage. To realize the contraction encirclement, **A** decays with **a** that decreases from 2 to 0. The prey is attacked through spiraling model when the food location is locked. At this time, the location search updating strategy of whales is shown as follows [40, 41]:

(9) $$\begin{array}{c} x\left(m+1\right)=x\wedge \left(m\right)+B\wedge •e^{bo}•\;\cos\left(2\pi o\right),\\ B\wedge =\left|x\wedge \left(m\right)-x\left(m\right)\right| \end{array}$$

where *b* (*b* = 1) as a constant is the spiral shape; *o* is a random number in the interval [−1, 1]; **B**∧ represents the distance between the whale and the locked food.

Assume that the probability of the whale taking the action of shrinking encirclement and spiral attack is 50%, and the position updating strategy is expressed as follows:

(10) $$\begin{array}{c} \left\{\begin{array}{c} x\left(m+1\right)=x\wedge \left(m\right)-A•B,\;p<0.5,\\ x\left(m+1\right)=x\wedge \left(m\right)+B\wedge •e^{bo}•\;\cos\left(2\pi o\right),\;p\geq 0.5, \end{array}\right. \end{array}$$

where *p* is a random number in the interval [0, 1].

In addition, whales randomly searching for food can succeed through updating **A**. The whale can search for food in a larger area when |*A*| > 1 and search for food in a smaller area when |*A*| < 1.

(11) $$\begin{array}{c} B=\left|C\cdot x_{\text{rand}}\left(m\right)-x\left(m\right)\right|, \end{array}$$

(12) $$\begin{array}{c} x\left(m+1\right)=x_{\text{rand}}\left(m\right)-A•B, \end{array}$$

where **x**_rand_ represents a random position vector.

In the WOA algorithm, most of the parameters are random, and only the maximum number of iterations and population size need to be set, which is one of the advantages of the algorithm.

### 2.3. EWOA Algorithm

Wolpert and Macready [42] believed that no optimization algorithm can solve all optimization problems according to the “no free lunch” theory. It means that different optimization algorithms may obtain different solutions under the same issue. Therefore, developing new algorithms may achieve better results. The traditional WOA algorithm may suffer from some disadvantages even it has stronger optimization capability than Particle Swarm Optimization (PSO) and differential evolution algorithms, etc. For example, its coefficient *a* decreases linearly to achieve shrinking encirclement, but the dynamic changes during the iteration process are not convincing. The population diversity is also limited in the later iteration, resulting in being trapped into local minimum. The EWOA model is thus developed to resolve above problems. First, the dynamic attenuation coefficient *d*_*a*_ is introduced to simulate the dynamic change situation in the shrinking and enveloping behaviors of whales during the iterative process. The mathematical model of the dynamic attenuation coefficient is defined as follows:

(13) $$\begin{array}{c} d_{a}=2*{\left(\frac{\left(m_{\max}-m\right)}{m_{\max}}\right)}^{3}, \end{array}$$

where *m*_max_ represents the maximum number of iterations and *m* is the current iteration coefficient.

The value of dynamic attenuation coefficient over iterations is depicted in Figure 1. It can be seen that the coefficient (*d*_*a*_) value declines faster in the initial stage of the iteration, which enables locking the food position shortly. During the later iteration period, it decays slower but strengths the algorithm's local exploration ability instead.

Aiming at the deficiency of population diversity weakening in the later iteration, an area search updating strategy is proposed. The whales migrate to other regions to search for food by the regional update frequency *M* during the optimization process. It can promise the population diversity reaching to a large extent, thus improving the algorithm's optimization ability. The whale's update position is shown as follows:

(14) $$\begin{array}{c} x\left(m+1\right)=\text{rand }n\left(0,\sigma^{2}\right)•x\left(m\right)+x\left(m\right), \end{array}$$

where rand *n*(0, *σ*^2^) obeys Gaussian distribution.

Similar to WOA algorithm, most parameters in EWOA algorithm are random, but the maximum number of iterations, population size, and migration frequency need to be set in advance.

The process flowchart of the EWOA algorithm for searching the global optima is shown in Figure 2.

As shown in Figure 2, EWOA algorithm optimization process includes the following steps:

1. Initialize EWOA algorithm parameters.
2. Determine whether to implement area search updating strategy.
3. If the area search updating strategy is implemented, the location is updated according to equation (14); otherwise the location is updated according to equations (10) and (12) [36].
4. Update the optimal location of whale population [37].
5. Determine whether to terminate the iteration. If the iteration is terminated, the optimization is completed. Otherwise, return to step (2).

### 2.4. Convergence Analysis

There are five standard test functions used to analyze the model convergence efficiency. The *f*_1_, *f*_2_, and *f*_3_ are unimodal functions, where the local extremum is the global optima, while *f*_4_ and *f*_5_ are multimodal functions. The variable ranges in functions are listed in Table 1.

In addition to EWOA algorithm, PSO algorithm [26], crow search algorithm (CSA) [27], and classic WOA algorithm were chosen tests for comparison. Note that CSA algorithm is a new type of swarm intelligence optimization algorithm with better convergence performance and is suitable as a comparison algorithm. PSO algorithm is a classic optimization algorithm and is usually used as a comparison algorithm. Simultaneously, the traditional WOA algorithm is used as a comparison algorithm to compare the convergence results with the EWOA algorithm. Algorithms' parameters are set as shown in Table 2.

In PSO, *w*_max_ and *w*_min_are the maximum and minimum values, respectively. *C*1 and *C*2 are the learning coefficients. In CSA, *AP* is the consciousness probability. *FL* is the flight length. *b* is used to define the spiral shape in both WOA and EWOA algorithms. *M* represents the search update frequency in EWOA. The population size is 30, and the maximum number of iterations is 500. The algorithms are tested under a unified platform, and each optimization algorithm is repeated 30 times for optimizing each test function. The average convergence value, the best convergence value, and the worst convergence value from every test function are concluded in Table 3.

As can be seen, the EWOA algorithm presents better search outcomes than others. Obviously, the results obtained from unimodal functions such as *f*_1_, *f*_2_, and *f*_3_ consistently outperform those of multimodal functions like *f*_4_ and *f*_5._ Furthermore, PSO and CSA algorithms showed poor optimization results in multimodal functions, where the worst value is up to 28.85 in PSO. For all unimodal functions, the WOA algorithm can achieve very low optimal value close to 0, while the EWOA algorithm reaches the optimal value, i.e., 0.

The fitness function to evaluate the convergence process is defined as follows:

(15) $$\begin{array}{c} \text{fitness}=\sqrt{\frac{\sum_{i=1}^{nn}{\left(P_{\text{train},i}-P_{\text{train},i}^{*}\right)}^{2}}{n}}, \end{array}$$

where *n* is the number of training samples; *P*_train*,i*_ represents the E-commerce transaction training value; and *P*_train,*i*_^*∗*^ indicates the E-commerce transaction prediction value.

The iterative convergence curves (log (Fitness)) using WOA and EWOA algorithms in various test functions are shown in Figure 3. The convergence speed of EWOA algorithm is considerably faster than WOA algorithm in all test functions, requiring much shorter iterations to converge.

## 3. Analysis of Multiple Influencing Factors in E-Commerce Transactions Trend

E-commerce transaction volume indicates the average value of E-commerce sales volume and E-commerce procurement volume. The E-commerce transactions sample set was collected from 2005 to 2019 in China, including the annual E-commerce transaction volume and the multiple influencing factors. The influencing factors in E-commerce transactions mainly consist of basic resource, transaction level, and economic development level. The basic resources include the Internet penetration rate (A1; unit: %), number of websites (A2; unit: ten thousand), number of CN domain names (A3, unit: ten thousand), and number of Internet users (A4; unit: 100 million). Indeed, the Internet penetration rate is to reflect the sharing degree of basic resources. Websites applied as a transaction platform are an important index on E-commerce transactions; the number of CN domain names can reflect the number of Internet service companies. The number of Internet users is to reflect the demand for shopping services via Internet.

In transaction level, the factors including express delivery business volume (A5; unit: 100 million) and express delivery business revenue (A6; unit: 100 million yuan) have a crucial impact on transactions level. Among them, express delivery business plays an important role in the E-commerce sales. On the other hand, the express delivery business revenue can reflect the level of E-commerce transactions in the express delivery industry. In economic development level, Gross Domestic Product (GDP) regarded as a macroeconomic factor is considered a key factor in the economic activity. It can reflect the situation of the E-commerce development. Therefore, GDP (A7; unit: trillion yuan) is used to evaluate the E-commerce transactions in this study.

The statistics on China's E-commerce transactions volume and the influence factors from 2005 to 2019 are presented in Table 4. It indicates that E-commerce transaction volume (*T*) increases every year, i.e., from 1.29 trillion in 2005 to 34.81 trillion in 2019. Similarly, other influencing factors, e.g., A1–A7, in E-commerce transactions have a growing trend, in which A5 and A6 increase much more than others.

The gray correlation is employed to analyze the correlation degree between multiple influencing factors and E-commerce transaction volume. Initially, the dimensionless process in E-commerce transaction volume and influencing factors is implemented to reduce the difference between the numerical values. Then, the correlation coefficient is calculated. The E-commerce transaction volume is denoted as the reference sequence {*x*_0_(*t*)}, and the influencing factors are denoted as the comparison subsequence {*x*_*i*_(*t*)}. The correlation coefficients at time k are expressed as follows. The difference (Δ_*i*_(*k*)) between the reference sequence {*x*_0_(*t*)} and the comparison sequence {*x*_*i*_(*t*)} is as follows:

(16) $$\begin{array}{c} \Delta_{i}\left(k\right)=\left|x_{0}\left(k\right)-x_{i}\left(k\right)\right|. \end{array}$$

The correlation coefficient *C*_*i*_(*k*) between the *i*_th_ comparison sequence and the reference sequence is as follows:

(17) $$\begin{array}{c} C_{i}\left(k\right)=\frac{\Delta_{\min}+0.5\Delta_{\max}}{\Delta_{i}\left(k\right)+0.5\Delta_{\max}}, \end{array}$$

where Δ_*i*_(*k*) represents the absolute difference between the two sequences at time *k*, Δ_min_ is the minimum absolute difference of the comparison sequences, and Δ_max_ is the maximum absolute difference of the comparison sequences.

The correlation degree (*cr*_*i*_) between the *i*_th_ comparison sequence and the reference sequence is defined in the following equation:

(18) $$\begin{array}{c} cr_{i}=\frac{1}{n}\sum_{k=1}^{n}C_{i}\left(k\right), \end{array}$$

where *n* denotes the number of the sequence data.

The correlation degree between E-commerce transaction volume and multiple influencing factors is presented in Table 5.

It reveals that the highest correlation degree in the express business revenue (A6) reaches 0.91; the correlation degrees in Internet penetration rate (A1), number of CN domain names (A3), and number of Internet users (A4) exceed 0.8; the correlation degrees in website number (A2), express delivery business volume (A5), and GDP (A7) are below 0.8. As above, the collected data from A1, A3, and A4, A6 are considered as the input variables for the forecasting models.

## 4. Model Implementation with Case Analysis

### 4.1. E-Commerce Transaction Prediction Using the EWOA-SVM Model

Based on the integration of EWOA and SVM models, the proposed EWOA-SVM model is established to forecast E-commerce transactions trend. The architecture of prediction process is depicted in Figure 4, being demonstrated as follows:

1. Analyze the impact of multiple influencing factors on E-commerce transaction volume
2. Calculate the correlation degree between different influencing factors and E-commerce transactions through gray correlation using equation (18)
3. Select strongly related factors with E-commerce transactions as model input variables
4. Classify the training set and test set, and normalize the data
5. Construct E-commerce transaction trend prediction model using EWOA-SVM
6. Set the parameters of EWOA algorithm and SVM model [40]
7. Train EWOA-SVM model using training set
8. Use EWOA to optimize the random parameters of SVM
9. Calculate the fitness values of EWOA algorithm through equation (15) [41]
10. Output the optimal parameters of SVM after the training process is complete
11. Verify EWOA-SVM model using test set
12. Employ trained SVM to predict E-commerce transaction trends
13. Evaluate the forecast results of E-commerce transaction

The performance of all algorithms throughout this study was carried out using MATLAB software, and the code of core programs and datasets can be freely accessed on the web page https://drive.google.com/drive/folders/1OPlt_W_u8XHrvT_PW-wOwUBZtUL2mind?usp=sharing.

The root mean square error (rmse) [46] and fitting coefficient *r*_2_ [47] are used to evaluate the model performance, where rmse represents the prediction error, and *r*_2_ indicates the changing trend of the predictive values. When the fluctuating trend of the predictive value is closer to the real one, the *r*_2_ is closer to 1.

(19) $$\begin{array}{c} \text{rmse}=\sqrt{\frac{1}{\text{num}}\sum_{i=1}^{\text{num}}{\left(P_{\text{test},i}-P_{\text{test},i}^{*}\right)}^{2}},\\ r_{2}=1-\frac{\sum_{i=1}^{\text{num}}{\left(P_{\text{test},i}-P_{\text{test},i}^{*}\right)}^{2}}{\sum_{i=1}^{\text{num}}{\left(P_{\text{test},i}-{\bar{P}}_{\text{test},i}\right)}^{2}}, \end{array}$$

where num is the number of testing samples; *P*_test*,i*_ is the test value of E-commerce transaction; *P*_test,*i*_^*∗*^ represents the predicted value of E-commerce transaction; and ${\bar{P}}_{\text{test},i}$ is the average test value of E-commerce transaction.

### 4.2. Case 1

Two cases were used to test the effectiveness of the proposed EWOA-SVM model, also including the SVM and WOA-SVM model for comparison. SVM model is selected to analyze the influence of random parameters on the prediction results, and WOA-SVM model is chosen to compare with the mining capability of the EWOA algorithm. The E-commerce transaction data collected from 2005 to 2014 was chosen as the training set, and the data collected between 2015 and 2019 was used as the test set. The training convergence curves in both WOA-SVM and EWOA-SVM models are presented in Figure 5. It indicates that the convergence speed of the EWOA algorithm is significantly faster than WOA algorithm. Moreover, the fitness value of the EWOA algorithm is obviously smaller than that of the WOA algorithm during the iteration process.

The test results from the performance of SVM, WOA-SVM, and EWOA-SVM models are presented in Figure 6. The specific prediction values are listed in Table 6. It is found that the prediction of WOA-SVM and EWOA-SVM models fits well with the actual E-commerce transaction curve. On the contrast, the SVM model shows a relatively higher error, particularly in 2015.

### 4.3. Case 2

The E-commerce transaction data collected between 2005 and 2010 was selected as the training set, and the data collected between 2011 and 2019 was used as the test set. The training convergence curves of the WOA-SVM and EWOA-SVM models are presented in Figure 7. It reveals that the convergence speed of the EWOA algorithm is faster than that of the WOA algorithm. Besides, the fitness value of the EWOA algorithm is considerably smaller than that of the WOA algorithm during iteration process. The results from the prediction performance of SVM, WOA-SVM, and EWOA-SVM models are shown in Figure 8. It indicates that the prediction accuracy of WOA-SVM and EWOA-SVM models is relatively higher than that of SVM model in general, well fitting with the actual E-commerce transactions trend. Nevertheless, the predicted result in SVM model is satisfactory except 2014 to 2015, showing more deviation from the actual values. The detailed prediction outcomes are listed in Table 7.

### 4.4. Evaluation of Test Results

The SVM, WOA-SVM, and EWOA-SVM models were used to predict the trend of E-commerce transactions in Cases 1 and 2. The prediction results of the model were evaluated in this section. For Cases 1 and 2, the relative error (Re%) curves from SVM, WOA-SVM, and EWOA-SVM models are shown in Figure 9, where the Re% values are concluded in Table 8.

For Case 1, the Re interval of the SVM model was [−9.61%, 1.23%]; the Re interval of the WOA-SVM model was [−2.75%, −2.98%]; the Re interval of the EWOA-SVM model was [−2.73%, 2.06%]. The fluctuation range of the EWOA-SVM model was the smallest, and the Re error of the model was significantly smaller than the other two models. For Case 2, the maximum Re value for WOA-SVM and EWOA-SVM exceeded 27%. The prediction error of E-commerce in 2013 was relatively large, but the remaining errors were less than 20%. The overall prediction effects of WOA-SVM and EWOA-SVM models were better than that of SVM model.

The prediction evaluation results using the rmse and *r*_2_ from the SVM, WOA-SVM, and EWOA-SVM models are listed in Table 9. In Case 1, the rmse values of WOA-SVM and EWOA-SVM models are contained below 0.6, where the minimum rmse value as 0.51 is obtained in EWOA-SVM model. It verifies that the rmse of EWOA-SVM model is 13.56%, 47.42% smaller than that of WOA-SVM and SVM models, respectively. However, the fitting result of the SVM model is better than others, showing its *r*_2_ value up to 99%. In Case 2, the rmse values in all three models significantly increase, being compared with Case 1. The minimum rmse of the EWOA-SVM model is 1.26, which is 14.86% and 17.64% smaller than that of the WOA-SVM and SVM models, respectively. Additionally, the EWOA-SVM model reaches the highest *r*_2_ value up to 98.42% among all models.

### 4.5. Discussion about Theory and Real Applications

At present, the global economy has entered a brand-new information network era. E-commerce is a new type of business operation model, which has been fast inspired with the impetus of the information technology. As E-commerce has the characteristics of wide transaction coverage, low cost, fast information circulation, and high work flow coordination, it has become a new engine for economic development. Accordingly, E-commerce transaction trend is becoming an important indicator to measure the business or economic activity level. To this end, this study proposes the EWOA-SVM model to predict the trend of E-commerce transactions, which provides a theoretical and effective tool for E-commerce development.

In real applications, a precise E-commerce transaction trend prediction can provide a decision-making basis for the governments or enterprises to formulate relevant development policies or plans in future business or industrial investments. The proposed model in this study can mine the crucial factors with high correlation degree in E-commerce transactions and construct E-commerce transaction trend correlation indexes. Importantly, it can be applied to logistics enterprises, Internet enterprises, and other information network companies in their business behavior.

## 5. Conclusions

In this study, the model training data was collected from E-commerce transactions volume and the influence factors, e.g., A1–A7, between 2005 and 2019. This sufficient data support and robust EWOA network structure can effectively alleviate the overfitting problem. The evaluation results of each model have been given more evidence with discussion to clarify this issue. The main contributions in this paper are concluded as follows:

1. A dynamic search coefficient and search updating strategy are combined to solve WOA algorithm's limitations. Accordingly, the EWOA algorithm can reach the global optima, i.e., 0, for multimodal functions, indicating a strong ability to escape from local minima.
2. The express delivery, Internet penetration rate, number of CN domain names, and number of Internet users are confirmed as the most crucial factors in the E-commerce transactions trend.
3. The evaluation results demonstrate that the EWOA-SVM model is superior to existing algorithms in the prediction of E-commerce transaction trend. For example, rmse of the EWOA-SVM model for Case 1 is 13.56% smaller than that of the WOA-SVM model and 47.42% smaller than that of SVM model. In Case 2, the rmse of the EWOA-SVM model is 14.86% smaller than that of the WOA-SVM and 17.64% smaller than that of the SVM model.

In the future work, it suggests that additional influencing factors in E-commerce transaction trend may be extended in practical circumstances. Besides, the generalization ability for various data prediction may be improved further.

## Figures and Tables

**Figure 1:** Dynamic attenuation coefficient over iterations.

**Figure 2:** Flowchart of EWOA optimization process.

**Figure 3:** Convergence curves of WOA and EWOA algorithms. (a) *f*_1_. (b) *f*_2_. (c) *f*_3_. (d) *f*_4_. (e) *f*_5_.

**Figure 4:** Flowchart of E-commerce transaction forecast.

**Figure 5:** Training convergence curves of WOA and EWOA algorithms between 2005 and 2014.

**Figure 6:** Test results of E-commerce transactions between 2015 and 2019.

**Figure 7:** Training convergence curves of WOA and EWOA algorithms between 2005 and 2010.

**Figure 8:** Test results of E-commerce transactions from 2011 to 2019.

**Figure 9:** Prediction error curves. (a) Prediction relative errors in Case 1. (b) Prediction relative errors in Case 2.

**Table 1:** Standard test functions and variable ranges [43–45].

Equations	Variable ranges	Global optima	dim
*f*_1_(*v*)=∑_*i*=1_^dim^*v*_*i*_^2^	[−100, 100]	0	30
*f*_2_(*v*)=∑_*i*=1_^dim^(∑_*j*=1_^*i*^*v*_*j*_)^2^	[−00, 100]	0	30
*f*_3_(*v*)=∑_*i*=1_^dim^|*v*_*i*_|+∏_*i*=1_^dim^|*v*_*i*_|	[−10, 10]	0	30
$f_{4}\left(v\right)=\left(1/4000\right)\sum_{i=1}^{\dim}v_{k}^{2}-\prod_{i=1}^{\dim}\cos\left(v_{i}/\sqrt{i}\right)+1$	[−600, 600]	0	30
*f*_5_(*v*)=10*∗*dim+∑_*i*=1_^dim^(*v*_*i*_^2^ − 10*∗* cos(2*πv*_*i*_))	[−5.12, 5.12]	0	30

Note: “dim” denotes the test dimension.

**Table 2:** Optimization algorithm parameters.

Algorithms	Parameters
PSO	*w*_max_ = 0.9; *w*_min_ = 0.3; *C*1 = *C*2 = 1.49
CSA	*AP* = 0.1; *FL* = 2
WOA	*b* = 1
EWOA	*b* = 1; *M* = 20

**Table 3:** Achievement of convergence results.

Test function	Algorithm	Average result	Best result	Worst result
*f*_1_	PSO	0.1083	5.51*e* − 07	2.41
	CSA	2.49*e* − 04	4.54*e* − 06	9.01*e* − 04
	WOA	1.49*e* − 72	6.38*e* − 85	4.34*e* − 71
	EWOA	1.51*e* − 266	8.82*e* − 313	4.52*e* − 265

*f*_2_	PSO	24.66	2.38*e* − 02	373.84
	CSA	0.16	2.70*e* − 03	1.75
	WOA	3.98*e* − 09	3.95*e* − 11	4.72*e* − 06
	EWOA	1.56*e* − 217	1.89*e* − 248	4.46*e* − 216

*f*_3_	PSO	0.81	4.98*e* − 02	3.09
	CSA	6.85*e* − 02	1.90*e* − 03	0.81
	WOA	5.54*e* − 51	7.70*e* − 59	1.01*e* − 49
	EWOA	1.50*e* − 154	2.38*e* − 173	4.49*e* − 153

*f*_4_	PSO	0.31	6.74*e* − 02	0.75
	CSA	0.17	4.79*e* − 02	0.47
	WOA	5.8*e* − 03	0	0.17
	EWOA	0	0	0

*f*_5_	PSO	15.52	7.96	28.85
	CSA	9.25	3.97	17.90
	WOA	3.78*e* − 15	0	5.68*e* − 14
	EWOA	0	0	0

**Table 4:** Statistics of E-commerce transactions.

Year	A1	A2	A3	A4	A5	A6	A7	*T*
2005	8.5	69.4	109	1.11	8.66	239.7	18.58	1.29
2006	10.5	84	180	1.37	10.6	299.7	21.76	1.54
2007	16	150	900	2.1	12.02	342.6	26.8	2.17
2008	22.6	287	1357	2.98	15.13	408.4	31.67	3.14
2009	28.9	323	1368	3.84	18.58	479	34.56	3.67
2010	34.3	191	435	4.57	23.39	574.6	40.89	4.55
2011	38.3	250	353	5.13	36.73	758	48.41	6.09
2012	42.1	255	751	5.64	56.85	1005.3	53.41	8.11
2013	45.8	320	1082	6.17	91.87	1441.7	58.8	10.4
2014	47.9	355	1129	6.48	139.59	2045.4	63.59	16.39
2015	50.3	425	1636	6.88	206.7	2760	68.9	21.79
2016	53.2	482	2061	7.51	313.5	4005	74.41	26.1
2017	55.8	533	2084	7.72	400.6	4957	82.07	29.16
2018	59.6	523	2124	8.29	507.1	6010	91.92	31.63
2019	61.2	518	2185	8.85	630	7450	99.08	34.81

Note: “*T*” represents E-commerce transaction volume (trillion yuan; 1 yuan≈0.15 USD).

**Table 5:** Gray correlation degree in various influencing factors.

Gray correlation degree (*cr*_*i*_)			
A1	0.81	A5	0.79
A2	0.79	A6	0.91
A3	0.85	A7	0.77
A4	0.81		

**Table 6:** Results of E-commerce transactions forecast from 2015 to 2019.

Year	Actual	SVM	WOA-SVM	EWOA-SVM
2015	21.79	19.69616	21.94652	21.73803
2016	26.1	25.92237	26.24643	26.63792
2017	29.16	28.82402	28.35714	28.36315
2018	31.63	32.02076	32.57347	32.20004
2019	34.81	34.98426	34.36644	34.55087

**Table 7:** Results of E-commerce transactions forecast from 2011 to 2019.

Year	Actual	SVM	WOA-SVM	EWOA-SVM
2011	6.09	5.923791	6.09362	6.322908
2012	8.11	8.275549	7.878242	6.545946
2013	10.4	11.43486	13.30829	13.27391
2014	16.39	14.07154	15.8526	16.24195
2015	21.79	18.59799	20.41689	21.19814
2016	26.1	24.75947	24.83894	25.52773
2017	29.16	27.97686	27.22712	27.7213
2018	31.63	31.79973	32.85884	32.54913
2019	34.81	35.85496	36.01635	35.09898

**Table 8:** Forecast error values.

Case	Year	Re (%)		
		SVM	WOA-SVM	EWOA-SVM
Case 1	2015	−9.61	0.71	−0.23
	2016	−0.68	0.56	2.06
	2017	−1.15	−2.75	−2.73
	2018	1.23	2.98	1.80
	2019	0.50	−1.27	−0.74

Case 2	2011	−2.72	0.10	3.82
	2012	2.04	−2.85	−19.28
	2013	9.95	27.96	27.63
	2014	−14.14	−3.27	−0.90
	2015	−14.64	−6.30	−2.71
	2016	−5.13	−4.83	−2.19
	2017	−4.05	−6.62	−4.93
	2018	0.53	3.88	2.91
	2019	3.01	3.46	0.83

**Table 9:** Evaluation results of each model.

Cases	Models	rmse	*r*_2_ (%)
Case 1	SVM	0.97	99.27
	WOA-SVM	0.59	98.23
	EWOA-SVM	0.51	98.69

Case 2	SVM	1.53	97.79
	WOA-SVM	1.48	98.30
	EWOA-SVM	1.26	98.42

## Data Availability

The data used to support the findings of this study are included within the article.
